# Chitinase 1 regulates pulmonary fibrosis by modulating TGF-β/SMAD7 pathway via TGFBRAP1 and FOXO3

**DOI:** 10.26508/lsa.201900350

**Published:** 2019-05-13

**Authors:** Chang-Min Lee, Chuan-Hua He, Jin Wook Park, Jae Hyun Lee, Suchita Kamle, Bing Ma, Bedia Akosman, Roberto Cotez, Emily Chen, Yang Zhou, Erica L Herzog, Changwan Ryu, Xueyan Peng, Ivan O Rosas, Sergio Poli, Carol Feghali Bostwick, Augustine M Choi, Jack A Elias, Chun Geun Lee

**Affiliations:** 1 Molecular Microbiology and Immunology, Brown University, Providence, RI, USA; 2 Department of Internal Medicine, Yonsei University College of Medicine, Seoul, South Korea; 3 Section of Pulmonary, Critical Care, and Sleep Medicine, Department of Internal Medicine, Yale School of Medicine, New Haven, CT, USA; 4 Brigham and Women’s Hospital, Boston, MA, USA; 5 Department of Medicine, College of Medicine, Medical University of South Carolina, Charleston, SC, USA; 6 Weill Cornell Medicine Pulmonary and Critical Care Medicine, New York, NY, USA; 7 Division of Medicine and Biological Sciences, Brown University, Warren Alpert School of Medicine, Providence, RI, USA

## Abstract

TGF-β1 is a critical mediator of tissue fibrosis in health and disease whose effects are augmented by chitinase 1 (CHIT1). However, the mechanisms that CHIT1 uses to regulate TGF-β1–mediated fibrotic responses have not been defined. Here, we demonstrate that CHIT1 enhances TGF-β1–stimulated fibrotic cellular and tissue responses and TGF-β1 signaling. Importantly, we also demonstrate that these effects are mediated by the ability of CHIT1 to inhibit TGF-β1 induction of its feedback inhibitor, SMAD7. CHIT1 also interacted with TGF-β receptor associated protein 1 (TGFBRAP1) and forkhead box O3 (FOXO3) with TGFBRAP1 playing a critical role in CHIT1 enhancement of TGF-β1 signaling and effector responses and FOXO3 playing a critical role in TGF-β1 induction of SMAD7. These pathways were disease relevant because the levels of CHIT1 were increased and inversely correlated with SMAD7 in tissues from patients with idiopathic pulmonary fibrosis or scleroderma-associated interstitial lung disease. These studies demonstrate that CHIT1 regulates TGF-β1/SMAD7 axis via TGFBRAP1 and FOXO3 and highlight the importance of these pathways in the pathogenesis of pulmonary fibrosis.

## Abstract (precis)

Chitinase 1 (CHIT1) plays a role in the pathogenesis of pulmonary fibrosis by modulating canonical and noncanonical TGF-β signaling via interaction with TGFBRAP1 and FOXO3. These findings highlight the CHIT1/SMAD7 axis as a potential biomarker and therapeutic target of pulmonary fibrosis.

## Introduction

TGF-β1 is a pleiotropic regulator of essential biologic responses (Massague, 1998). Central to its biology are its well-documented roles in wound healing and its importance as a regulator of inflammation, and cell survival, differentiation, motility, proliferation, and adhesion (Bowen et al, 2013). TGF-β1 dysregulation has been implicated in the pathogenesis of a wide variety of diseases and is a potent regulator of scarring in human diseases characterized by fibrogenesis (Bowen et al, 2013). In many of these disorders, the overexpression of TGF-β1 has been documented. In other diseases, such as scleroderma (SSc), exaggerated levels of TGF-β1 are not seen, but TGF-β1 signatures are appreciated (Sargent et al, 2010). In keeping with its multifaceted effector functions and complex roles in health and disease, it is now clear that the production and effector responses of TGF-β1 are under precise control (Bowen et al, 2013). The factors that regulate TGF-β1 effector response, however, have not been adequately defined.

The GH 18 gene family contains true chitinases that bind and cleave chitin. Chitinase 1 (CHIT1, chitotriosidase) is the most readily appreciated true chitinase in mammals and man. It can be found in the circulation and tissues of normal controls and patients with disorders characterized by inflammation and remodeling such as Gaucher’s disease, sarcoidosis, chronic obstructive pulmonary disease, and interstitial pulmonary fibrosis (Cho et al, 2015). However, its roles in these disorders are poorly understood because chitin (the only known substrate of chitinases) does not exist in mammals. Previous studies from our laboratory demonstrated that the levels of CHIT1 activity are increased in patients with SSc with interstitial lung disease (SSc-ILD) where they correlate with disease severity (Lee et al, 2012). In vivo and in vitro investigations also demonstrated that CHIT1 interacted with TGF-β1 to augment TGF-β1 receptor–induced SMAD and MAPK and AKT signaling (Lee et al, 2012). These studies demonstrate that CHIT1 is a biomarker for TGF-β1 in SSc-ILD where it augments TGF-β1 signaling (Lee et al, 2012). However, the mechanism(s) by which these fibrogenic effects of CHIT1 are mediated have not been adequately defined.

The effects of TGF-β1 ligands are mediated by type 1 and type 2 receptors (Huang & Chen, 2012). They activate and phosphorylate receptor-regulated SMAD proteins (SMAD2 and 3), which form a heterometric complex with SMAD4. The complexes then translocate to the nucleus where it regulates gene expression and activates canonical and noncanonical signaling pathways (Miyazawa & Miyazono, 2017). In keeping with the critical importance of the regulation of TGF-β1 effector responses, TGF-β1 signaling is regulated by a variety of inhibitory mechanisms (Miyazawa & Miyazono, 2017). Inhibitory SMADs, in particular SMAD7, are induced by TGF-β1 and feedback to control TGF-β1 signaling responses (Yan et al, 2009; Sureshbabu et al, 2016). In addition to TGF-β1, a variety of other cytokines and microRNA regulate SMAD7. However, a relationship between CHIT1 and SMAD7 has not been defined.

To further understand the mechanisms that CHIT1 uses to regulate TGF-β1 response, in vivo and in vitro approaches were used to define the roles of CHIT1 and the mechanisms that it uses in pulmonary fibrosis. These studies demonstrate that CHIT1 augments TGF-β1–stimulated fibroblast proliferation, myofibroblast differentiation, and canonical and noncanonical signaling. They also demonstrate that these responses are mediated by the ability of CHIT1 to inhibit SMAD7 via interaction with TGF-β receptor–associated protein 1 (TGFBRAP1) and FOXO3. Last, they highlight the disease relevance of these findings by demonstrating the increased levels of CHIT1 and decrease in SMAD7 in lung tissues from patients with idiopathic pulmonary fibrosis (IPF) or SSc-ILD.

## Results

### CHIT1 enhances TGF-β1–stimulated fibroblast responses in vitro

To determine if CHIT1 has significant effects on the TGF-β1–stimulated cellular responses that could contribute to fibrosis, we stimulated normal human lung fibroblasts (NHLFs) with recombinant (r) CHIT1 alone, or in combination with TGF-β1. CHIT1 by itself did not stimulate fibroblast proliferation, but it did enhance TGF-β1–stimulated fibroblast proliferation as measured by WST-1 assay (Fig 1A). Similarly, CHIT1 did not alter fibroblast differentiation into myofibroblasts as assessed by α-smooth muscle actin (α-SMA) accumulation, but it augmented the ability of TGF-β1 to enhance α-SMA accumulation (Fig 1B). This suggests that CHIT1 enhances TGF-β1–stimulated myofibroblast transformation. In accord with these findings, TGF-β1 stimulated the expression of vimentin, paxicillin, fibronectin, and other extracellular matrix (ECM) genes such as elastin and collagen, and these effects were significantly enhanced by CHIT1 (Fig 1C). Collectively, these results indicate that CHIT1 enhances TGF-β1–stimulated fibroblast proliferation, myofibroblast transformation, and ECM expression.

**Figure 1.** CHIT1 enhances TGF-β1-stimulated fibroblast responses in vitro. NHLF were stimulated with recombinant (r) TGF-β1 (rTGF-β, 10 ng/ml) and rCHIT1 (250 ng/ml) for 24 h then the effect of rTGF-β and rCHIT1 was evaluated. **(A)** Fibroblast cell proliferation assay by WST-1. **(B)** Immunohistochemistry (IHC) using anti–α-smooth muscle actin; Con, controls with no rTGF-β or rCHIT1 stimulation. **(C)** Expression of markers of myofibroblasts and extracellular protein accumulation assessed by real-time quantitative reverse transcription PCR (qRT-PCR). β-actin was used as an internal control. The values in panels A and C represent mean ± SEM of triplicated evaluations in a minimum of two separate experiments. Panel B is a representative IHC in a minimum of three separate experiments. *P < 0.05, **P < 0.01, *t* test. Bars in panel B, 50 μM.

### CHIT1 enhances and plays a critical role in TGF-β1–stimulated fibrotic responses in vivo

Studies were next undertaken to determine if CHIT1 influenced TGF-β1–induced fibrotic responses in vivo. In these experiments, we first compared the regulation of ECM proteins in transgenic mice in which CHIT1 and TGF-β1 were overexpressed in the lungs, individually or in combination. We also compared the effects of transgenic TGF-β1 in mice with wild-type or null mutant CHIT1 alleles. In accord with our in vitro findings cited above, although transgenic or null mutation of CHIT1 alone did not stimulate or suppress, transgenic TGF-β1 was a significant stimulator and CHIT1 and TGF-β1 interacted to further stimulate the expression of ECM proteins, including fibronectin, elastin, and type 1 collagen (Fig 2A). Importantly, the ability of TGF-β1 to stimulate ECM proteins was at least partially dependent on CHIT1 because the stimulatory effects of transgenic TGF-β1 were significantly decreased in mice with null CHIT1 loci (Fig 2B and C). When viewed in combination, these studies demonstrate that CHIT1 is both necessary and sufficient for optimal TGF-β1–stimulated fibrotic ECM tissue response in the lungs.

**Figure 2.** CHIT1 enhances and plays a critical role in TGF-β1–stimulated signaling and fibrotic responses in vivo. 6–8-wk-old WT (−), TGF-β Tg (+), *Chit1* Tg (+), and *Chit1 Tg*/TGF-β Tg mice were subjected to the evaluation. These mice were euthanized after 14 d of transgene induction of doxycycline containing drinking water (0.5 g/l). The expression levels of TGF-β1 and Chit1 in the bronchoalveolar lavage measured ELISA were about 1.8 ± 0.2 ng/ml and 13 ng ± 2.3/ml for TGF-β Tg and Chit1 Tg, respectively. **(A, B)** Evaluation on the ECM-associated gene expression and collagen accumulation in the lungs of WT and TGF-β Tg mice with overexpression of Chit1 (*Chit1* Tg) (A) or null mutation of Chit1 (*Chit1*^*−/−*^) (B) using real-time qRT-PCR or Sircol Collagen Assay. β-actin was used as an internal control. **(C)** Representative Mallory’s trichrome staining of the lungs from TGF-β Tg mice with null mutation of Chit1 (*Chit*^*−/−*^). **(D, E)** Western blot analysis on the activation of TGF-β signaling (MAPK/Erk, Akt and, and Smad2) and Smad7 expression using lung lysates from WT and TGF-β and *Chit1* Tg mice. β-actin was used as an internal control. The values in panels A and B represent the mean ± SEM of five mice each group. Panels D and E are representative Western blots in a minimum of three separate experiments. *P < 0.05, **P < 0.01, ***P < 0.001, *t* test. Bars in panel C, 100 μm.

### CHIT1 augments TGF-β signaling in the lung

Studies were next undertaken to define the role(s) of CHIT1 in TGF-β signaling. In these experiments, we compared the activation of canonical TGF-β1 signaling pathways in the lungs from transgenic mice in which CHIT1 and TGF-β1 were targeted to the lung, alone and in combination. This approach was undertaken because previous studies from our laboratory highlighted the exaggerated fibrotic responses in the lungs from mice in which CHIT1 and TGF-β1 were simultaneously expressed compared with mice in which each was expressed individually (Lee et al, 2012). As can be seen in Fig 2D, the present studies demonstrated that transgenic TGF-β1 increased canonical Smad2/3, MAPK/Erk, and Akt activation compared with wild-type control mice and activation of these signaling pathways was further enhanced in the co-expression of TGF-β1 and Chit1. These studies demonstrate that CHIT1 augments TGF-β1 signaling in vivo.

### CHIT1 inhibits the expression of inhibitory SMAD7

TGF-β1 is well known to induce SMAD7 which, in turn, feeds back to control TGF-β1 signaling and effector responses (Zhao et al, 2000). The studies described above demonstrate that CHIT1 augments TGF-β1 signaling and fibrotic responses. This led us to hypothesize that the effects of CHIT1 might be mediated via alterations in the ability of TGF-β1 to induce SMAD7. To test this hypothesis, we compared the expression of Samd7 in in the lungs from transgenic mice in which Chit1 and TGF-β1 were expressed, alone and in combination. In these experiments, transgenic TGF-β1 was a potent stimulator, and transgenic Chit1 did not significantly alter the expression of Smad7 (Fig 2E). Importantly, when Chit1 and TGF-β1 were simultaneously overexpressed, the ability of TGF-β1 to stimulate Samd7 was markedly ameliorated (Fig 2E). These studies demonstrate that CHIT1 inhibits the ability of TGF-β1 to induce inhibitory SMAD7. In so doing, they support the concept that the synergistic interactions of CHIT1 and TGF-β1 are mediated, at least in part, by the ability of CHIT1 to inhibit the SMAD7-mediated feedback inhibition that normally controls TGF-β1 response.

### CHIT1 interacts with TGFBRAP1 and FOXO3

Studies were next undertaken to further define the mechanisms that CHIT1 uses to regulate TGF-β1 signaling and cell and tissue responses. Because CHIT1 is a secreted protein that can be found in both extracellular and intracellular compartments, we first undertook studies to define its potential binding partner(s). Potential CHIT1-binding partners were first defined using yeast 2 hybrid (Y2H) screening assays with a lung cDNA library. This approach identified several CHIT1-binding proteins, including TGFBRAP1 and FOXO3 (Table S1). TGFBRAP1 has been reported to be a chaperone for SMAD signaling (Wurthner et al, 2001) and FOXO3 is an transcription factor for multiple genes that play critical roles in metabolism, cellular stress response, tissue remodeling, and disease progression (Nho & Hergert, 2014; Webb et al, 2016). In keeping with their potential importance, the results of the Y2H assays were further evaluated using co-immunoprecipitation (Co-IP) and co-localization assays. The Co-IP and immunoblot evaluations of cells transfected with CHIT1, TGFBRAP1, and FOXO3 demonstrated significant molecular interactions between CHIT1 and TGFBRAP1 or FOXO3 (Fig 3A). The molecular interaction between CHIT1 and TGFBRAP1 or FOXO3 was further supported by the co-localization immunohistochemical evaluations on the NHLF after stimulation with recombinant TGF-β (Fig 3B). We noted similar pattern of CHIT1 expression and co-localization with TGFBRAP1 or FOXO3 in epithelial cells and macrophages (data not shown). When viewed in combination, these studies demonstrate that CHIT1 interacts with TGFBRAP1 and FOXO3.

Table S1 CHIT1 interacting proteins detected by yeast-2 hybrid analysis.

**Figure 3.** CHIT1 interacts with TGFBRAP1 and FOXO3. **(A)** Co-immunoprecipitation (IP) and immunoblot (IB) evaluations on the MLE12 epithelial cells transfected with CHIT1, TGFBRAP1, and FOXO3 expressing constructs. **(B)** Double-labeled fluorescent IHC to localize expression of CHIT1, TGFBRAP1, and FOXO3 in NHLF. Panels A and B are representative Western blots and IHC evaluations of three separate experiments, respectively. Bars in panel B, 50 μm.

### TGFBRAP1 plays a critical role in CHIT1 augmentation of TGF-β1 signaling

To define the role(s) of TGFBRAP1 in CHIT1 regulation of TGF-β signaling, gene-specific siRNA silencing was used. In these experiments, NHLF cells were stimulated with rTGF-β1 (10 ng/ml) and rCHIT1 (250 ng/ml), alone and in combination, for 1 h. Comparisons were made of cells treated with TGFBRAP1 siRNA (which decreased the levels of TGFBRAP1 protein expression by >75%, Fig 4A) or scrambled controls. As noted above, the simultaneous treatment of fibroblasts with recombinant CHIT1 with TGF-β1 enhanced the ability of TGF-β1 to activate SMAD2 and MAPK/ERK and AKT. Importantly, these CHIT1-stimulated TGF-β1 responses were markedly decreased in cells treated with TGFBRAP1 siRNA (Fig 4A). We also noted modest decreases in TGFβR1 expression with TGFBRAP1 silencing, suggesting that Chit1 regulates TGF-β receptor expression via TGFBRAP1, at least in part. Luciferease-tagged SMAD2 promotor assay further confirmed that silencing of TGFBRAP1 ameliorate the CHIT1-induced promoter activity of SMAD2 with TGF-β stimulation (Fig 4B). Collectively, these studies indicate that TGFBRAP1 plays an essential role in the ability of CHIT1 to augment canonical and noncanonical TGF-β1 signaling and TGFβR expression.

**Figure 4.** TGFBRAP1 plays a critical role in CHIT1 augmentation of TGF-β1 signaling and TGFβR expression. **(A)** Western blot evaluation on the NHLF cells stimulated by rTGF-β and/or rCHIT1 with (+) and without (−) siRNA silencing of TGFBRAP1. Scrambled siRNA was used as control for TGFBRAP1 specific siRNA. **(B)** Evaluation on the SMAD activities on the cells transfected SMAD2-luciferase construct after stimulated by rTGF-β (20 ng/ml) and/or rCHIT1 (100 or 200 ng/ml) with and without siRNA silencing of TGFBRAP1. Panel A is a representative immunoblot of three separate experiments. Values in panel B represent the mean ± SEM of triplicated evaluations in a minimum of two separate experiments. *P < 0.05, **P < 0.01, one-way ANOVA.

### TGF-β1 stimulates SMAD7 via FOXO3

The studies noted above demonstrate that CHIT1 interacts with FOXO3, and we identified a FOXO3-binding site in the promoter region of SMAD7. This led us to investigate whether FOXO3 plays a role in TGF-β1 and or CHIT1’s regulation of SMAD7 expression. In these experiments, NHLF cells were treated with TGF-β1 and rCHIT1, alone or in combination, with and without siRNA silencing of FOXO3. The siRNA that were used in these experiments decreased the levels of FOXO3 by >70% (Fig S1). As noted above, TGF-β1 treatment increased SMAD7 mRNA expression in a manner that was reduced by the simultaneous administration of CHIT1 (Fig 5A). In these experiments, the silencing of FOXO3 reduced TGF-β1–stimulated SMAD7 expression to the levels comparable with those seen in control cells (Fig 5A). The role of FOXO3 in TGF-β1–stimulated SMAD7 expression was further validated using SMAD7 promoter-luciferase assays. In these experiments, HEK293 cells were transfected with SMAD7 promoter-luciferase constructs that contain a wild-type FOXO3 consensus sequence (ProSMAD7^WT^) (GTAAAC, located −802 bp upstream of SMAD7 translation initiation site) (Fig S2) and SMAD7 luciferase activity was evaluated after treatment with recombinant TGF-β1 and CHIT1, alone or in combination. As shown in Fig 5B, TGF-β1 stimulated SMAD7 luciferase activity in a manner that was opposed by co-administration of rCHIT1. As can also be seen in Fig 5B, this stimulation was SMAD7-dependent because SMAD7 luciferase activity was not induced by TGF-β1 in cells that had been transfected with a mutant SMAD7 promoter construct (ProSMAD7^▽(Foxo)^), which did not contain a FOXO3 consensus sequence. When viewed in combination, these studies demonstrate that the transcription factor FOXO3 plays a critical role in TGF-β1 stimulation of SMAD7 expression.

**Figure S1.** FOXO3 siRNA Silencing efficacy on NHLFs. NHLFs were treated with scrambled control siRNA (scrambled) and Foxo3-specific siRNA (FOXO3 SiRNA), and then the expression of FOXO3 was evaluated using qRT-PCR after 24-h incubation. RPL13a was used as internal control. n = 3 each group. Values represent the mean ± SEM of triplicated evaluations. **P < 0.01, *t* test.

**Figure 5.** TGF-β stimulates SMAD7 expression via FOXO3. **(A)** Real-time qRT-PCR evaluations on the NHLF cells after stimulation with rTGF-β (10 ng/ml) and rCHIT1 (250 ng/ml) with (+) and without (−) siRNA silencing of FOXO3. **(B)** HEK293 cells transfected with luciferase-tagged SMAD7 promoter construct with (ProSMAD7^WT^; WT) and without (ProSMAD7^▽(FOXO3)^; mutant form) FOXO3 consensus sequence were stimulated with rTGF-β and/or rCHIT1, and then luciferase activity was measured. **(C)** Western blot evaluations on the pFOXO3 and FOXO3 expression in the lungs of WT (−), TGF-β Tg (+), CHIT1 Tg (+), and CHIT1/TGF-β Tg mice. Whole-lung lysates were further separated into cytoplasmic and nuclear fractions and subjected to the immunoblots using anti-pFOXO3 and FOXO3 antibodies. Values in panels A and B represent the mean ± SEM of triplicated evaluations in a minimum of two separate experiments. Panel C is a representative immunoblot of three separate experiments. H3, histone H3, used as internal control of nuclear protein. **P < 0.01, ***P < 0.001, one-way ANOVA. ns, not significant.

**Figure S2.** Generation of deletion mutant of FOXO consensus sequence. FOXO consensus sequence (GTAAACA) located 802 bp upstream of SMAD7-coding region was deleted using site-directed mutagenesis (ProSMAD7^▽(Foxo)^) and compared with wild-type promoter of SMAD7 (ProSMAD7^WT^).

### CHIT1 reduces the levels of TGF-β–stimulated nuclear FOXO3/pFOXO3

Our studies demonstrate that TGF-β1 stimulates SMAD7 via FOXO3, whereas CHIT1 inhibits TGF-β1–stimulated SMAD7. This led us to determine if the inhibitory effects of CHIT1 could be attributed to its ability to regulate FOXO3. To address this issue, we evaluated the expression of Foxo3 and pFoxo3 in whole-cell lysates and the cellular nuclear and cytoplasmic fractions from the cells of lungs from WT mice and mice in which TGF-β1 and or Chit1 were targeted to the lungs. As shown in Fig 5C, transgenic TGF-β1 modestly increased the levels of Foxo3 and pFoxo3 in the whole-lung lysates and their nuclear and cytoplasmic fractions. Although transgenic Chit1 did not significantly alter the expression of Foxo3 and pFoxo3 by itself, it did increase the levels of TGF-β1–stimulated Foxo3 or pFoxo3 in the whole-lung lysates (Fig 5C). This was mainly due to a significant increase in cytoplasmic Foxo3 and pFoxo3 with decreased nuclear fraction of these moieties (Fig 5C). These studies demonstrate that CHIT1 regulates the ability of TGF-β1 to induce the nuclear transcription factor FOXO3 and suggests that CHIT1 inhibits TGF-β1 induction of SMAD7 by decreasing nuclear FOXO3 accumulation.

### The levels of CHIT1 expression are increased in IPF where they correlate inversely with SMAD7

Studies were next undertaken to determine if our murine findings are relevant to patients with IPF. Because CHIT1 augmented TGF-β1–induced fibrotic tissue responses by inhibiting SMAD7, we characterized the expression of CHIT1 and SMAD7 in tissues and cells from IPF patients and normal controls. As shown in Fig 6A, the levels of mRNA encoding CHIT1 were significantly higher in the lungs from patients with IPF compared with normal controls. In accord with our murine studies, there was an inverse correlation between the levels of expression of SMAD7 and CHIT1 in the IPF patients (Fig 6B). To further investigate the interactions between these moieties, alveolar epithelial cells (alveolar type 1 [AT1] + alveolar type 2 cells [AT2]) were isolated from controls and IPF patients, and the levels of mRNA encoding CHIT1 and SMAD7 were characterized. These evaluations revealed increased levels of expression of CHIT1, decreased levels of SMAD7 expression, and an inverse correlation between the expression of CHIT1 and SMAD7 in cells from IPF patients (Fig 6 C–E). Interestingly, when AT1 and AT2 cells were evaluated separately, CHIT1 and SMAD7 were similarly regulated (Fig S3). As seen in our murine modeling systems, these studies demonstrate that, CHIT1 is up-regulated in patients with IPF where its expression correlates inversely with the expression of SMAD7.

**Figure 6.** Increased expression levels of CHIT1 in the patients with IPF where they correlate inversely with SMAD7. **(A)** Real-time qRT-PCR evaluations on the expression levels of CHIT1 in whole-lung lysates from normal controls and IPF patients. **(B)** A scatter plot with regression analysis demonstrating inverse relationship between the levels of CHIT1 and SMAD7 expression in the lungs of IPF patients (Spearman rank test, *P* = 0.04). **(C, D)** qRT-PCR evaluations on CHIT1 and SMAD7 expression in alveolar epithelial cells (alveolar type 1 epithelial cells [AT1] and alveolar type 2 epithelial cells [AT2]) isolated from the lungs of normal controls and IPF patients. **(E)** A scatter plot with regression analysis demonstrating inverse relationship between the levels of CHIT1 and SMAD7 in alveolar epithelial cells isolated from the lungs of IPF patients (*P* = 0.036, Spearman’s rank test).

**Figure S3.** Expression levels of CHIT1 and Smad7 in the lung epithelial cells from the patients with IPF and controls. The expression levels of CHIT1 and SMAD7 in alveolar type 1 (AT1) and type 2 (AT2) cells detected by qRT-PCR, respectively. *P < 0.01, *t* test.

### Decreased SMAD7 expression in the lungs from patients with SSc-ILD

Previous studies from our laboratory, demonstrated that the levels of CHIT1 activity in the circulation of patients with SSc-ILD are increased where they correlate with abnormal lung function (Lee et al, 2012). To determine if the murine and IPF findings noted above are also relevant to SSc-ILD, we also evaluated the expression of SMAD7 in tissues from these patients and determined if the levels of CHIT1 activity correlated with disease progression. As can be seen in Fig 7A and B, the levels of expression of SMAD7 were decreased in lungs from patients with SSc-ILD when compared with controls. In addition, the levels of circulating CHIT1 activity were increased in the patients with progressive SSc-ILD compared with stable SSc-ILD (Fig 7C), and overall progression-free survival was decreased in patients with increased levels of CHIT1 activity in a manner that persisted even after adjustment for the relevant covariates of age, gender, race, and smoking status (Fig 7D). These findings demonstrate that CHIT1 is induced, whereas Samd7 is inhibited in SSc-ILD and support the concept that the CHIT1/SMAD7 axis plays a critical role in the development and progression of pulmonary fibrosis in SSc-ILD.

**Figure 7.** Decreased SMAD7 expression in the lungs from patients with SSc-ILD. **(A)** IHC evaluation on the SMAD7 expression in the lung sections from normal control and patients with SSc-ILD. SMAD7 staining of SSc-ILD lungs (right) reveals decreased number of Samd7-positive cells especially in the stromal region as compared with normal control (left) that showed a number of parenchymal cells and also macrophages are strongly stained. **(B)** Quantitation of SMAD7-positive (+) cells in the lung sections from controls and SSc-ILD per high-powered field. **(C)** Serum CHIT1 activity in the SSc-ILD patients with stable and progressive lung function. “Progressive” was defined in the patients with more than 10% of absolute drop of forced vital capacity (FVC). **(D)** Survival analysis based on the levels of chitinase activity (below and above median value of 53.54 nM/ml/h) in the patients with SSc-ILD. SSc-ILD subjects (n = 56) with values exceeding the median value of 53.54 (dotted line) demonstrate reduced progression-free survival as defined by absolute loss of %FVC within 2 years of enrollment. Scale bars, 30 μm, **P < 0.01, ***P < 0.001, Spearman’s rank test. n, number of individuals subjected to the evaluation.

## Discussion

Although mammals do not have chitin or chitin synthase, substantial levels of chitinases and chitinase-like proteins are noted in the circulation as well as in local tissues (Lee et al, 2009, 2011; Cho et al, 2015). CHIT1, a major enzymatically active true chitinase, is produced, stored, and secreted by macrophages and neutrophils (van Eijk et al, 2005) and plays important roles in innate immune homeostasis (Elias et al, 2005). This can be appreciated in the pivotal roles it plays in host defenses against chitin-containing pathogens such as fungi, protozoa, and insects (Boot et al, 2001). As a sensitive biomarker of macrophage activation, dysregulated expression of CHIT1 in the circulation or local tissue has been reported in a variety of human diseases, including Gaucher’s disease, diabetes, sarcoidosis, inflammatory bowel disease, atherosclerosis, Alzheimer’s disease, and prostate cancer (Kanneganti et al, 2012; Elmonem et al, 2016). Recent studies from our laboratory and others also demonstrated that CHIT1 is dysregulated in lung diseases characterized by inflammation and remodeling such as bacterial infection, asthma, chronic obstructive pulmonary disease, and pulmonary fibrosis (Lee et al, 2012; Cho et al, 2015; James et al, 2016; Hong et al, 2018; Sharma et al, 2018). However, the specific mechanisms that CHIT1 uses to contribute to the pathogenesis of specific disease have not been fully understood. This is particularly true for CHIT1 in pulmonary fibrosis. Although we reported an important role of CHIT1 in the pathogenesis of SSc-ILD, however, the exact mechanism that CHIT1 uses to regulate pulmonary fibrosis has not been determined and the relevance to other forms of ILD remains uncertain.

In this study, we demonstrated that CHIT1 synergistically enhances TGF-β–stimulated fibroblast proliferation and myofibroblast transformation, and CHIT1 is sufficient and necessary for optimal TGF-β–stimulated ECM deposition in the lungs. We identified TGFBRAP1 and FOXO3 as interacting partners of CHIT1 that regulate TGF-β signaling and effector functions. Our studies further demonstrated that CHIT1 enhances TGF-β–stimulated activation of SMAD2/3, AKT, and MAPK/ERK pathways mainly through TGFBRAP1 while inhibiting the expression of SMAD7, a prototype of inhibitory SMAD of TGF-β signaling, via interaction with FOXO3. In support of these findings, we also noted increased expression of CHIT1 in the lungs or circulation of the patients with IPF or SSc-ILD, and the levels of CHIT1 were inversely correlated with SMAD7 expression in the lungs of these patients. When viewed in combination, these studies demonstrated a significant role of CHIT1 in the pathogenesis of pulmonary fibrosis via regulation of canonical and noncanonical TGF-β–stimulated signaling and SMAD7 expression.

IPF, a prototypic fibrotic disorder, is a progressive lung disease characterized by epithelial damage, fibroproliferative matrix deposition, and parenchymal remodeling (Raghu, 1998; Selman et al, 2001; Krein & Winston, 2002). TGF-β is believed to play an important role in this dysregulation because it is expressed in an exaggerated fashion in IPF where, in contrast to controls, a sizable percentage is biologically active (Khalil et al, 1996, 2001; Xu et al, 2003). The important role that TGF-β may play in this disorder can be seen in studies that demonstrate that TGF-β is a critical mediator of pulmonary fibrosis after bleomycin injury (Nakao et al, 1999; Yehualaeshet et al, 2000) and that transgenic overexpression in the lung or high-dose adenoviral TGF-β1 transfer causes progressive pulmonary fibrosis in vivo (Sime et al, 1997; Kelly et al, 2003; Lee et al, 2004) and IPF-like fibroblastic foci in in vitro explants (Xu et al, 2003). It is also interesting to note that TGF-β requires other cofactors that activate or enhance TGF-β signaling in the development of persistent fibrosis in the lung or other organs (Mori et al, 1999; Leask, 2006; Tatler & Jenkins, 2012). In this regard, present studies support a possibility that CHIT1 could be the one that enhances the signaling and effector function of TGF-β in the development of pulmonary fibrosis. In the previous studies, we demonstrated that overexpression of IL-13 induced prominent pulmonary fibrosis with increased expression of both TGF-β and CHIT1 (Lee et al, 2012). We also demonstrated that null mutation of CHIT1 without direct intervention of TGF-β significantly reduced IL-13–induced pulmonary fibrosis, suggesting a critical role of CHIT1 in TGF-β effector function in tissue fibrosis (Lee et al, 2012). Collectively, these findings suggest that CHIT1 plays an essential role in the pathogenesis of pulmonary fibrosis in which CHIT1 and TGF-β are dysregulated. In this regard, it is reasonable to speculate that CHIT1 also could play an important role in the pathogenesis of other organ fibrosis including sarcoidosis and nonalcoholic steatohepatitis that showed dysregulated levels of both CHIT1 and TGF-β (Peverill et al, 2014; Casanova et al, 2015).

Recently, Van Dyken et al (2017) reported that acidic mammalian chitinase (AMCase) plays a protective role in spontaneously developed pulmonary fibrosis related to chitin polymer accumulation in the lung. AMCase and CHIT1 are two true chitinases in mammals and have different cellular and tissue expression and physiologic function, although they share similar chitinolytic enzyme activity with different reaction conditions. It has been shown that AMCase, but not CHIT1, is prominently expressed in the murine lung, whereas the expression of Chit1 (both in endogenous and induced expression) is predominant in human lungs (Boot et al, 2005). Because the physiologic role of AMCase in the lungs is more likely adapted to the chitin-rich environment, it is reasonable to speculate that decreased chitinase activity of AMCase in murine lung results into chitin accumulation. However, in human lungs, there is no endogenous source of chitin, and CHIT1 enzyme activity was reported to be increased with ageing (Kurt et al, 2007) and in the lungs of IPF (Bargagli et al, 2007). These studies suggest that enzymatic deficiency of AMCase may not fully explain human lung pathologies without simultaneous consideration of Chit1, the major true chitinase expressed in human lungs. In addition, recent studies also support a direct pathogenic role of chitinase-like proteins such as CHI3L1 that have no chitinase enzyme activity with retained chitin-binding ability, in tissue remodeling and fibrosis (Zhou et al, 2014, 2015). These studies suggest that enzyme activity of either AMCase or CHIT1 might not be the sole responsible factor for determining final outcome of tissue response associated with chitinase dysregulation. When viewed in combination, present studies suggest that the relative contribution and potential interaction of AMCase and CHIT1 in the pathogenesis pulmonary fibrosis need to be further determined in future studies.

In this study, we demonstrate that CHIT1 interacts with intracellular proteins TGFBRAP1 or FOXO3 and regulates major TGF-β signaling and SMAD7 expression. As a chaperone for SMAD4, TGFBRAP1 has been shown to associate with inactive heteromeric TGF-β and activin receptor complexes, mainly through the type 2 receptor, and is released upon activation of signaling and recruit SMAD4 to the vicinity of the receptor complex to facilitate its interaction with receptor-regulated SMADs, such as SMAD2 (Wurthner et al, 2001). However, the specific role of TGFBRAP1 in the pathogenesis of fibrosis in the lungs or other organs has not been studied. This is the first study showing TGFBRAP1 interacts with CHIT1 and mediates synergistic effect of CHIT1 on TGF-β–stimulated canonical and noncanonical signaling. It is also interesting to note that silencing of TGFBRAP1 itself on normal lung fibroblasts minimally alters the TGF-β activation of SMAD2 or MAPK/ERK, but CHIT1 effects on these TGF-β signaling activation were abrogated, suggesting that TGFBRAP1 is a fine tuner of TGF-β signaling and effector function in the lung. It is also interesting to note that there is modest decrease in the expression of TGFβR1 expression with silencing of TGFBRAP1, suggesting that CHIT1 regulates TGF-β receptor expression via TGFBRAP1, at least in part.

Because silencing of TGFBRAP1 did not alter CHIT1 inhibition of TGF-β–stimulated SMAD7 expression, we sought other mechanism(s) responsible for CHIT1 regulation of SMAD7 expression. Our studies demonstrated that FOXO3, a transcriptional factor that has a binding consensus sequence in the promoter region of SMAD7, plays a critical role in TGF-β and CHIT1-regulated expression of SMAD7. TGF-β itself induced the expression and phosphorylation of both cytoplasmic and nuclear FOXO3. Interestingly, CHIT1 increases the levels of pFOXO3 in the cytoplasmic compartment with depletion pFOXO3 in nuclear fraction. These studies suggest that CHIT1 plays a role in nuclear/cytoplasmic shuttling and cytoplasmic retention of pFOXO3, which might limit the accessibility of FOXO3 in the nuclear fraction, resulted into decreased transcriptional activity of FOXO3 for SMAD7 or other FOXO3 target genes. Because our studies show that FOXO3 is essential for the expression of SMAD7, these results provide a potential mechanism to explain the inverse relationship between the levels of CHIT1 and SMAD7 expression noted in the lungs of IPF patients. In the previous studies, fibroblasts established from the patients with IPF showed that pathologic alteration of FOXO3 with reduced expression contribute to the progression of IPF by protecting fibroblasts from apoptotic or autophagic cell death responses (Im et al, 2015; Nho et al, 2011, 2013). It has been shown that Akt phosphorylation of FOXO3 resulted into nuclear cytoplasmic transport, and subsequent ubiquitination of this phosphorylated form of FOXO3 after binding with 14-3-3 protein is the major pathway of lowering FOXO3 levels in the fibroblasts or other cells (Kato et al, 2006; Tzivion et al, 2011; Im et al, 2015). A recent study also reported a critical role of FOXO3 in fibrogenesis and reduced expression of FOXO3 was implicated in the pathogenesis of IPF (Al-Tamari et al, 2018). Thus, current data are consistent with these findings in the sense that CHIT1 could contribute to the progression of pulmonary fibrosis via alteration of nuclear FOXO3 levels. However, the mechanism of CHIT1 regulation of cytosolic retention of pFOXO3 is not clear yet. Because increased levels of CHIT1 in fibrotic lungs of bleomycin-challenged mice were noted mainly in the cytoplasmic and perinuclear area of the cells (Fig S4), it is intriguing to speculate that physical binding between CHIT1 and pFOXO3 could be a reason for enhanced cytoplasmic retention of this moiety in the lung. It is also possible that CHIT1 uses other mechanism of pFOXO3 regulation such as interaction with 14-3-3 protein that facilitates the nuclear/cytosolic shuttling of pFOXO3 (Tzivion et al, 2011). These possibilities remain to be determined in the future studies.

**Figure S4.** Intracellular localization of Chit1 expression in the bleomycin-stimulated lung. Fluorescent IHC to localize Chit1 and early endosomal (EEA1) or lysosomal markers (Lamp1) on the lung tissue sections from bleomycin-challenged lungs. Open arrow, macrophage; closed arrow, type 2 alveolar epithelial cells; and yellow arrows, type 1 epithelial cells. **(A, B)** Bars in (A) and (B), 12 and 7 μm, respectively.

SMAD7, a major inhibitory SMAD of TGF-β signaling, blocks the function of SMAD2 and SMAD3 by inhibiting their binding to the activated receptors and exerting its negative effects on TGF-β1/SMAD signaling (Kavsak et al, 2000; Wang et al, 2016). The specific antifibrotic regulatory role of SMAD7 in the pathogenesis of pulmonary fibrosis has been demonstrated in various conditions. SMAD7 is the target of microRNAs associated with myofibroblast differentiation and bleomycin-induced lung fibrosis (Liu et al, 2010; Wang et al, 2016) and mediates IL-7 suppression of pulmonary fibrosis (Huang et al, 2002). In this regard, present studies provide CHIT1 as a novel negative regulator of SMAD7, which enhances TGF-β signaling and effector function.

It is interesting to note that dysregulated CHIT1 activity in the serum was significantly associated with progressive SSc-ILD compared with stable cases and that the levels of CHIT1 activity were correlated with survival rates of the patients. In the evaluation of end stage lungs from IPF patients, we also see prominent increases of CHIT1 expression with suppression of SMAD7 expression. These studies suggest that CHIT1/SMAD7 axis plays an important role in disease progression or exacerbation rather than initiator of fibrotic tissue response, and potential use of CHIT1/SMAD7 activity and expression both in serum and lung or BAL as a biomarker to predict disease severity and prognosis of patients with IPF and SSc-ILD.

In conclusion, these studies demonstrated that CHIT1 interacts with TGFBRAP1 and FOXO3 and enhances TGF-β–stimulated activation of canonical and noncanonical signaling and the expression of inhibitory SMAD7. Thus, CHIT1 and its interacting partners of TGFBRAP1 or FOXO3 could be reasonable therapeutic targets for the intervention of patients with pulmonary fibrosis in that TGF-β and CHIT1 are significantly dysregulated.

## Materials and Methods

### Mice

C57 BL/6 mice were purchased from the Jackson Laboratory and were housed at Brown University animal facilities. TGF-β Tg, *Chit1*^*−/−*^, and *Chit1* Tg mice on C57 BL/6 background were generated and maintained in our laboratory as previously described (Lee et al, 2004, 2012). Both TGF-β Tg and *Chit1* Tg mice are lung-specific inducible transgenic mice, and transgene expression was induced by drinking water containing doxycycline (0.5 g/l). The mice with null mutation or overexpression of Chit1 did not show any apparent abnormal phenotypes and developmental and signaling issues. All murine procedures were approved by the Institutional Animal Care and Use Committees at Brown University.

### Cell culture

NHLF cells and human embryonic kidney 293 cells (HEK293) were obtained from Lonza and American Type Culture Collection (ATCC), respectively. NHLF cells were cultured in fibroblast growth medium (Lonza CC-2512B) at 37°C in 5% CO_2_. HEK293 cells were maintained in DMEM supplemented with 10% FBS and 100 U/ml penicillin and 100 μg/ml streptomycin at 37°C in 5% CO_2_ incubator. NHLF cells were used within 10 passages according to the manufacturer's recommendation. MLE12 murine-transformed lung epithelial cells were purchased from ATCC and cultured and maintained using DMEM-F12 medium supplemented with 10% FBS as recommended.

### siRNA silencing of TGFBRAP-1 and FOXO3

siRNAs specific for human TGFBRAP1 (SC-36720; Santa Cruz) and FOXO3 (SC-37887; Santa Cruz) were used for silencing the levels of mRNA encoding TGFBRAP1 and FOXO3 as per the manufacturer’s instructions. NHLF cells were seeded on six-well plates and transfected the next day with TGFBRAP1, FOXO3, or control siRNAs. The cells were collected at the indicated time points and were subjected to real-time (RT)-PCR or Western blot evaluations.

### Co-IP and IB analysis

To assess interactions among CHIT1, TGFBRAP-1, and FOXO3, MLE12 murine lung epithelial cells were co-transfected with TGFBRAP1 and FOXO3 plasmids (pcDNA3.1). Lysates from these cells were subjected to immunoprecipitation using anti-hCHIT1 mouse monoclonal antibody (1/500 dilution, AF3559, R&D system). The Catch and Release V2.0 (Reversible Immunoprecipitation System; EMD Millipore) kit was used for Co-IP according to the manufacturer’s instruction. The precipitates were then evaluated by immunoblotting with antibodies against CHIT1, TGFBRAP1, or FOXO3.

### Co-localization with double-label IHC

To localize the expression of CHIT1, TGFBRAP1, and FOXO3, double-label IHC was undertaken with a modification of procedures described previously by our laboratory (Lee et al, 2016). NHLF cells (1 × 10^6^ cells/well) were cultured overnight in four-well chamber slides (Falcon) at 37°C in 5% CO_2_ incubator, then washed with PBS. To unmask antigens, the slides were placed for 20 min at high temperature under high pressure in citrate buffer (10 mM sodium citrate, 0.05% Tween 20, pH 6). The slides were then blocked with a nonserum protein-blocking reagent (DakoCytomation Inc) for 1 h at room temperature and incubated with primary antibodies (anti-CHIT1 [1/50 dilution, AF-5325; R&D system], anti-TGFBRAP1 [1/50 dilution, SC-13134; Santa Cruz Biotechnology], and anti-FOXO3 [1/50 dilution, 12829S; Cell Signaling]) for 60 min at room temperature in a humid chamber. Substitution of the primary antibody with PBS served as a negative control. The slides were then washed in PBST (0.01% Tween 20) and incubated with secondary antibodies conjugated with horseradish peroxidase (Cell Signaling). Reaction products were developed using DAB containing 0.3% hydrogen peroxide up to 5 min. Cell nuclei were stained with mounting medium with DAPI (50 μl, H-1200; Vector Laboratories). Fluorescence was detected by Immunofluorescence microscopy.

### Evaluation of TGF-β signaling

Canonical SMAD activity of TGF-β1 signaling pathway was assessed using dual reporter assays (SABiosciences). A SMAD-responsive firefly luciferase construct that constitutively expressed Renilla luciferase was transfected into NHLF cells. After stimulation with recombinant CHIT1 and TGF-β1, alone or in combination, SMAD activation was assessed by measuring the dual luciferase activities. SMAD2 activation and MAPK/ERK, AKT activation were evaluated by Western blot as previously described (Lee et al, 2004). The expression of SMAD7 was evaluated by immunoblot assay using anti-SMAD7 polyclonal rabbit antibody (Santa Cruz Biotechnology).

### Evaluation of FOXO3 and SMAD7 interaction

HEK293 cells were seeded at a density of 1 × 10^6^ cells/well in six-well dishes and grown to 70% confluence. For each well, 1 μg of pEZX-PG04-SMAD7 promoter construct (GeneCopoeia, Inc.) or 1 μg of the FOXO3-binding site point-mutated SMAD7 promoter were transfected into the cells with the Lipofectamine 3000 transfection reagent. After stimulation with rCHIT1 and rTGF-β1, alone or in combination, SMAD7 expression was assessed by measuring the Secrete-Pair Dual Luminescence Assay kit (GeneCopoeia, Inc.) and was normalized with secreted alkaline phosphatase activity within each sample.

### Evaluation on the levels of cytosolic and nuclear pFOXO3 and FOXO3

Phosphorylation and cytoplasmic/nuclear shuttling are the major pathways regulating transcriptional activity of FOXO3 (Nho & Hergert, 2014). Hence, studies are undertaken to see whether CHIT1 is implicated in this process. For this evaluation, cytosolic and nuclear fraction of the whole-lung lysates were prepared using nuclear cytoplasmic extraction reagents (Thermo Fisher Scientific) according to the procedures provided by the company and subjected to immunoblot evaluation using anti-pFoxO3 (Serine253) (Cell Signaling) and FoxO3 (D19A7) (Cell Signaling).

### Profiling of IPF and control lung tissues

Fresh human lung tissue was procured from subjects with end-stage lung disease, undergoing transplant or donor lungs that were not implanted at the time of transplant. The demographics and clinical characteristics of the groups can be seen in Table S2. All protocols were approved by the Partners Institutional Review Board. For each subject, small pieces (<5 mm) of whole-lung tissue were treated with RNAlater (QIAGEN) and snap-frozen in liquid nitrogen before storage at −80°C.

Table S2 Demographic feature of IPF patients and controls used in this study.

### Isolation of alveolar epithelial cell type 1 and type 2

Fresh human lung explants were sliced and washed with cold sterile PBS. Visible airway structures, vessels, blood clots, and mucin were removed. Lung specimens were minced mechanically into small pieces (<1 mm^3^) and then incubated for 45 min in 37°C in modified medium containing DMEM/F12 with added digestion enzymes: Liberase thermolysin medium (Roche), elastase (EC-134; Elastin Products Company), and DNase I (Thermo Fisher Scientific). Digested tissue was filtered using a metal strainer. 10% FBS were added to the flow-through to stop the enzymatic reaction. The pellet was resuspended in DMEM/F12 medium and filtered using a 100-μm strainer. The cells were resuspended in freezing medium (10% FBS and 10% DMSO in DMEM/F12), aliquoted, and stored in liquid nitrogen. Thawed single-cell suspension was sorted using FACS. Sorting gate for AEC type 1 and type 2 were designed as follows: DAPI−/CD45−/EpCAM+/PDPN+ and DAPI−/CD45−/EpCAM+/PDPN−, respectively. Isolated cells from 10 subjects diagnosed with IPF and 10 controls were used. Patient demographics and clinical information can be found in Table S3.

Table S3 Baseline demographics of a patient cohort and controls used to isolate AEC type 1 and type 2 cells.

### Cohort of SSc-ILD patients

These studies were performed with HIC approval at the Yale School of Medicine. Samples from subjects with SSc-ILD according to current EULAR/ACR criteria were used for these studies. As shown in Table S4, subjects with CHIT1 levels exceeding the median level of 52.39 nM/ml/h were more likely to be older and to have smoked but were otherwise matched for gender, race, disease subtype, and lung function.

Table S4 Demographic feature of SSc patients and controls used in this study.

### Measurement of CHIT1 activity

CHIT1 enzyme activity was assessed as described previously in our laboratory (Lee et al, 2012).

### Localization of SMAD7 expression in SSc

IHC was undertaken to localize SMAD7 protein using polyclonal rabbit anti human SMAD7 obtained from Santa Cruz Biotechnology as described in our laboratory (Lee et al, 2009). Lung explants from patients with SSc-ILD and nonfibrotic controls were subjected to the staining and SMAD7 expressing cells were counted in six randomly chosen high power fields. The values averaged and the mean ± SEM calculated for SSc-ILD versus normal lung.

### Statistical analysis

Normality of data was assessed using the D’Agostino–Pearson omnibus normality test. Normally distributed data are expressed as the means ± SEM and assessed for significance by a *t* test or ANOVA, as appropriate. Categorical variables were compared using the Fisher’s exact test. Nonparametric correlation between two variables was evaluated by Spearman’s rank test.

## Supplementary Material

Reviewer comments
